The article "The impact of aqueous and N-hexane extracts of three Fabaceae species on seed germination and seedling growth of some broadleaved weed species" was retracted in 2022. Reasons: compromised peer review; a conflict of interest; concerns about the authorship.

# The impact of aqueous and N-hexane extracts of three Fabaceae species on seed germination and seedling growth of some broadleaved weed species

**DOI:** 10.1371/journal.pone.0258920

**Published:** 2021-11-05

**Authors:** Muhammad Ehsan Safdar, Xiukang Wang, Mudasar Abbas, Cumali Ozaslan, Muhammad Asif, Muhammad Adnan, Ali Tan Kee Zuan, Wenqiang Wang, Kristina Gasparovic, Omaima Nasif, Mohammad Javed Ansari

**Affiliations:** 1 Department of Agronomy, College of Agriculture, University of Sargodha, Sargodha, Pakistan; 2 College of Life Science, Yan’an University, Yan’an, China; 3 Faculty of Agriculture, Department of Plant Protection, Dicle University, Diyarbakir, Turkey; 4 Faculty of Agriculture, Department of Land Management, Universiti Putra Malaysia, UPM Serdang, Selangor, Malaysia; 5 Institut of Plant and Environmental Sciences, Slovak University of Agriculture, Nitra, Slovakia; 6 Department of Physiology, College of Medicine and King Khalid University Hospital, King Saud University, Medical City, Riyadh, Saudi Arabia; 7 Department of Botany, Hindu College Moradabad (Mahatma Jyotiba Phule Rohilkhand Univesity Bareilly), Moradabad, India; Ghazi University, PAKISTAN

## Abstract

Weed infestation is a persistent problem for centuries and continues to be major yield reducing issue in modern agriculture. Chemical weed control through herbicides results in numerous ecological, environmental, and health-related issues. Moreover, numerous herbicides have evolved resistance against available herbicides. Plant extracts are regarded as an alternative to herbicides and a good weed management option. The use of plant extracts is environmentally safe and could solve the problem of herbicide resistance. Therefore, laboratory and wire house experiments were conducted to evaluate the phytotoxic potential of three Fabaceae species, i.e., *Cassia occidentalis* L. (Coffee senna), *Sesbania sesban* (L.) Merr. (Common sesban) and *Melilotus alba* Medik. (White sweetclover) against seed germination and seedling growth of some broadleaved weed species. Firstly, N-hexane and aqueous extracts of these species were assessed for their phytotoxic effect against lettuce (*Lactuca sativa* L.). The extracts found more potent were further tested against germination and seedling growth of four broadleaved weed species, i.e., *Parthenium hysterophorus* L. (Santa-Maria), *Trianthema portulacastrum* L. (Pigweed), *Melilotus indica* L (Indian sweetclover). and *Rumex dentatus* L. (Toothed dock) in Petri dish and pot experiments. Aqueous extracts of all species were more toxic than their N-hexane forms for seed germination and seedling growth of lettuce; therefore, aqueous extracts were assessed for their phytotoxic potential against four broadleaved weed species. Aqueous extracts of all species proved phytotoxic against *T*. *portulacastrum*, *P*. *hysterophorus*, *M*. *indica* and *R*. *dentatus* and retarder their germination by 57, 90, 100 and 58%, respectively. Nevertheless, foliar spray of *C*. *occidentalis* extract was the most effective against *T*. *portulacastrum* as it reduced its dry biomass by 72%, while *M*. *alba* was effective against *P*. *hysterophorus*, *R*. *dentatus* and *M*. *indica* and reduced their dry biomass by 55, 68 and 81%, respectively. It is concluded that aqueous extracts of *M*. *alba*, *S*. *sesban* and *C*. *occidentalis* could be used to retard seed germination of *T*. *portulacastrum*, *P*. *hysterophorus*, *M*. *indica* and *R*. *dentatus*. Similarly, aqueous extracts of *C*. *occidentalis* can be used to suppress dry biomass of *T*. *portulacastrum*, and those of *M*. *alba* against *P*. *hysterophorus*, *R*. *dentatus*. However, use of these extracts needs their thorough testing under field conditions.

## Introduction

Weeds exist everywhere and obstruct the germination, growth, and yield of field crops. Furthermore, weeds compete with crop plants and suppress their growth by releasing different allelochemicals [1–3]. Weeds are a global threat for the sustainability of natural and agro-ecosystems [4]. Weeds are grouped as grasses, broadleaved and sedges. Weeds are categorized as wasteland and cropland weeds based on their infested habitats. Wasteland weeds emerge near agricultural fields, roadsides and railway tracks and do not directly obstruct crop production. Cropland weeds usually grow within cropping areas and interfere with crops for inputs and natural resources [5]. It is estimated that weeds cause 20–30% yield losses in major crops of Pakistan [6]. Weeds cause 35–69% yield losses in mungbean [7], 15–40% in cotton [8], 58–85% in soybean [9] and up to 40% in most of the field crops [10–12].

Herbicides are the most effective and quickest weed management option; however, they reduce food quality and impose many adverse effects on environment, animal and human health [13,14]. Furthermore, extensive use herbicides with same mode of action can result in the evolution of herbicide resistance [11,12]. Herbicide resistance has been confirmed in 304 weed biotypes in 95 crops from 71 countries, affecting efficiency of herbicides with 21 modes of action [15]. Therefore, environmental pollution and herbicide resistance problems forced the scientists to develop alternative weed management methods [16–18]. Utilization of the extracts derived from different plants has gained popularity as an alternative weed management option since last two decades [2,3,19,20]. These extracts have a significant potential to retard or promote seed germination and seedling growth of various weed species and the phenomenon is termed as allelopathy [1,21]. It is known that plant extracts leave less contamination and are more bio-degradable than synthetic herbicides [22]. Hence, phytochemicals derived from different plants can be utilized to control weeds [19,23,24]. These allelochemicals are released by plant parts in ecosystem through roots exudation, leaching, decomposition and volatilization of plant parts [19,23,24].

*Trianthema portulacastrum* L., *Parthenium hysterophorus* L., *Melilotus indica* L. and *Rumex dentatus* L. are broadleaved obnoxious weed species that are widely distributed throughout Pakistan [25]. Yield losses caused by these weed species in various crops may reach up to 30% by *T*. *portulacastrum* [26], 53% by *P*. *hysterophorus* [27], 45% by *M*. *indica* [28] and 83% by *R*. *dentatus* [29]. The use of plant extracts as an alternative weed management option has been proved successful for controlling many weed species. Bajwa et al. [30] reported complete inhibition of germination and seedling growth of *Avena fatua* L. with the application of extracts derived from *Cuscuta reflexa*, *Salvia moocraftiana* and *P*. *hysterophorus*. Likewise, Safdar et al. [31] demonstrated that leaf extracts of *Achyranthes aspera* L. and *Alternanthera philoxeroides* (Mart.) Griseb. inhibited seed germination and seedling growth of *P*. *hysterophorus*. Aqueous leaf extracts of *Artemisia absinthium* and *Psidium guajava* inhibited the seed germination, seedling growth of *P*. *hysterophorus* [32].

Many plants of Fabaceae have been explored for their allelopathic effect and proved effective against several weed species [33]. Zahir et al. [34] reported that *C*. *fistula* has strong allelopathic potential against numerous weed species. Yellow sweet clover contains coumarin, which is a most active allelopathic compound and can be used as a natural herbicide because of its high inhibitory effect on other plant species. There are some plants abundantly distributed in Soon Valley of district Khushab, Pakistan. These include *C*. *occidentalis* (coffee senna), *Sesbania sesban* (Egyptian riverhemp) and *Melilotus alba* (Yellow sweet clover). *Cassia occidentalis* is a woody plant and can grow during long days. This is an annual plant with rapid growth habit [35]. It has a great ability to inhibit growth of neighboring plants and has been found allelopathic against *P*. *hysterophorus* [33]. *Sesbania sesban* is a thin crowned, single or multi-stemmed, deep-rooted shrub or small sized tree which have 7 to 9 m height [36]. The plant rapidly grows up to 4.5 to 6.0 m in one year and its flowers develop into mature pods one year after germination [37]. *Melilotus alba* has 0.3–2.6 m height, upright stem, coarse or fine, ground or channeled usually pubescent or has piles near the tip [38]. Lettuce (*Lactuca sativa*) is considered highly sensitive to allelopathic action of phytotoxic compounds; therefore, widely used as target species in preliminary screening of allelopathic plants [39]. Members of Fabaceae family have rarely been explored for their allelopathic potential against broadleaved weed species. Different solvents like water, methanol, acetone, chloroform, ethyl acetate and hexane are being used for preparing plant extracts that vary in their allelochemical composition [40]. Previous studies have reported differential response of weeds to phytotoxicity of aqueous and N-hexane plant extracts [41–43].

This study explored phytotoxic activity of *Cassia occidentalis*, *Sesbania sesban* and *Melilotus alba* against seed germination and seedling growth of four weed species, i.e., *R*. *dentatus*, *P*. *hysterophorus*, *M*. *indica* and *T*. *portulacastrum*. It was hypothesized that N-hexane and aqueous extracts of these plant species may differ in their phytotoxicity against lettuce germination and subsequently against targeted weed species.

## Materials and methods

### Experiment details and sampling site

Both experiments were executed at College of Agriculture, University of Sargodha, Pakistan during 2 019 and 2020. The Sargodha lies at 72.69°E longitude and 32.07°N latitude, while Fabaceae plants were collected during the months of September and October 2018 from different Soon Valley sites, district Khushab, Pakistan. The sampling was done randomly from every location having maximum indigenous species diversity of selected family. There are no permits required for plant sampling at the collection site and species are not considered endangered or regulated as quarantine pests in the country.

### Preparation of plant extracts

Collected plant samples were packed in plastic bags and labelled with sample number, common or local name, location, and collection date. Afterwards, samples were carefully washed with distilled water to remove any contamination. Fine powder of samples (separately for each sample) was made through grinding in an electric blender. Grinding process was done with full care to avoid any impurities and mixing. The powder of every sample was weighed and packed in sealed plastic zipper bags. The extraction was done through Soxhlet and rotary evaporator. For the extraction, N-hexane was used as a solvent. The measured quantity of every powdered sample was placed in thimble and plugged with cotton. Afterwards, thimble was separately placed in Soxhlet apparatus and flask was filled with N-hexane (500 ml of solvent). Each sample was in Soxhlet apparatus for 4–6 hours. Samples were individually transferred to rotary evaporator for the final extraction. In rotary evaporator, solution was separated into the solvent and refined form of extracts were obtained. The extracts were kept in air-tight in black glass containers and stored in refrigerator for further use. For preparation of aqueous extracts, 5 g powder of each plant species was soaked in 100 mL distilled water for 24 h at room temperature [44] and then filtered through muslin cloth.

### Experiment 1. Phytotoxic effect of N-hexane and aqueous extracts of Fabaceae plants on seed germination of lettuce

A laboratory bioassay was carried out for preliminary screening of N-hexane and aqueous extracts of *Cassia occidentalis* (L.), *Sesbania sesban* (L.) Merr., and *Melilotus alba* Medik. on seed germination of lettuce (*Lactuca sativa* L.). There were two factors, i.e., plants extract [distilled water treated control (DWTC), *Cassia occidentalis* extract, *Sesbania sesban* (L.) Merr. extract and *Melilotus alba* Medik. extract] and extraction methods, i.e., A = Aqueous and N = N-hexane.

A filter paper (10 cm diameter) was placed in pre-washed and dried Petri dishes. Subsequently, 3 ml of all plant extracts was added to each dish. Twenty seeds of lettuce were placed in each dish. Consequently, Petri dishes were packed in the polythene bags to avoid moisture loss. The experiment was carried out at room temperature.

### Experiment 2: Phytotoxic effect of Fabaceae plants on seed germination and seedling growth of broadleaved weeds

This experiment evaluated phytotoxic effects of aqueous extracts of *Cassia occidentalis* (L.), *Sesbania sesban* (L.) Merr., and *Melilotus alba* Medik. on seed germination and seedling growth of parthenium (*Parthenium hysterophorus* L.), horse purslane (*Trianthema portulacastrum* L.), sweet clover (*Melilotus indica* L.) and toothed dock (*Rumex dentatus* L.). Distilled water was applied as control.

Twenty seeds were placed in sterilized Petri dishes having round discs of filter paper as described above. Extracts were applied and dishes were sealed with paraffin. For seedling growth plants were grown in plastic pots of 250 ml volume. Soil was taken from College of Agriculture, University of Sargodha. Soil was thoroughly mixed with sand at 1:1 ratio. Afterwards, 3–4 seeds of each weed species were sown in pot and pots were irrigated. The aqueous extracts were sprayed by hand sprayer on seedlings at 2–4 leaf stage. Second spray was done after five days of first spray. The data related to chlorophyll contents, dry weight (mg), seedling vigor index, leaf area (cm^2^), root and shoot length (cm) were taken.

### Data collection

Seed germination percentage (GP) was recorded by counting the germinated seeds on each day for 20 days. Seeds were considered germinated when growing plumule extended to length of about 2 mm, respectively. The GP was calculated by Eq 1 given by Association of Official Seed Analysts [45].


$$Germination\;percentage\;(\%)=\frac{Germinated\;seeds\;}{Total\;seeds}\times 100$$ (1)

Germination index (GI) w was calculated by Eq 2 given by Association of Official Seed Analysts [45].


$$GI=\frac{Number\;of\;germinated\;seeds}{Days\;of\;first\;count}+\frac{Number\;of\;germinated\;seeds}{Days\;of\;final\;count}$$ (2)

Time to obtain 50% germination (T_50_) was calculated according to Eq 3 devised by Coolbear et al. [46].


$$T_{50}=\mathrm{ti}+\frac{(\frac{N}{2}‐n_{i})\left(t_{j}‐t_{i}\right)}{n_{j}‐n_{i}}.$$ (3)

Where “N” represents the number of final germinated seeds whereas “nj” and “ni” are the cumulative number of germinated seeds by contiguous counts at times “tj” and “ti” respectively, where ni N/2 nj.

Seedling vigor index (SVI) was calculated by using Eq 4 given by Orchard [47].


SVI=Germinationpercenatge×Seedlinglength (4)

Germination energy (GE) is the ratio of germinated seeds at 4^th^ day of sowing to the total number of emerged seeds till 15^th^ day. It was determined by using Eq 5 proposed by Ruan et al. [48].


$$GE=\frac{Number\;of\;seeds\;germinated\;till\;4th\;day\;of\;sowing\;}{Total\;number\;of\;germinated\;seeds\;till\;15th\;day}$$ (5)

Three seedlings were randomly selected and their root and shoot lengths were measured and averaged. All seedlings from each Petri dish or pot were taken and wrapped in tissue paper and placed in oven at 70°C for 48 hours and then weighed on electric balance. Chlorophyll contents of three plants were determined with the help of chlorophyll meter (Yaxin, 1260) and average. Three plants from each treatment were chosen and washed. Afterwards, their leaf area was determined with the help of leaf area meter in cm^2^.

### Statistical analysis

First experiment was laid out according to randomized complete block design with factorial arrangement, while second experiment was laid out in completely randomized design and all treatments were replicated four times. Data were analyzed statistically using Fisher’s Analysis of Variance (ANOVA) technique (two-way for first experiment and one-way for second experiment) and treatment means were compared at 5% significance level by least significant difference post hoc test [49]. Normality in the data was tested by Shapiro-Wilk normality test and variables with non-normal distribution were normalized by Arcsine transformation technique. All statistical analysis were done on SPSS statistical software version 21 [50].

## Results

### Experiment 1

Data of various germination and seedling growth parameters of lettuce in response to aqueous and N-hexane extracts of plant species proved that aqueous extracts of all Fabaceae plants were phytotoxic for lettuce germination and growth (data not shown). Among Fabaceae plants, *M*. *alba* and *C*. *occidentalis* extracts showed the highest phytotoxicity against seed germination and seedling growth of lettuce.

### Experiment 2

Data regarding seed germination percentage of four broadleaved weed species in response to aqueous extracts of Fabaceae plants is given in Tables 1 and 2. Different extracts significantly altered the seed germination of tested weed species. The *M*. *alba* plant extract exhibited the highest inhibitory effect on seed germination of *T*. *portulacastrum* (31.25%), while *S*. *sesban* and *M*. *indica* reduced seed germination of *P*. *hysterophorus* by 6.25 and 0.00%. However, *C*. *occidentalis* extract reduced seed germination of *R*. *dentatus* by 26.2%.

**Table 1:** Analysis of variance (mean squares) of phytotoxic effect of aqueous plant extracts of *Fabaceous* plants on germination and seedling growth of different broadleaved weed species.

SOV	DF	GP	T_50_	GE	GI	RL	SL	SVI	DW
***T*. *portulacastrum***									
**Treatment**	3	1427.0***	3.62	443.7	50.15*	2.58***	4.48***	134718***	32.70***
**Error**	12	13.54	1.71	63.54	5.04	0.02	0.02	377	0.276
**Total**	15								
***P*. *hysterophorus***									
**Treatment**	3	2247.4**	2.16	1162.5***	424.3***	0.186***	2.18***	49652.2***	18.77
**Error**	12	250.5	6.10	51.04	16.56	0.026	0.078	1957.3	20.43
**Total**	15								
***R*. *dentatus***									
**Treatment**	3	1370.8***	2.36*	522.9***	122.7***	0.274***	0.970***	34149.8***	28.43***
**Error**	12	30.21	0.79	35.4	4.73	0.003	0.075	675.1	0.3654
**Total**	15								
***M*. *indica***									
**Treatment**	3	3008.3***	46.51***	143.7***	98.88***	80.82***	4.46***	97359.0***	33.35***
**Error**	12	91.67	0.723	17.70	3.80	57.72	0.115	3737.4	0.1413
**Total**	15								

SOV = source of variation

* = Significant, DF = degree of freedom, GP = germination percentage, T_50_ = time to 50% germination, GE = germination energy, GI = germination index, RL = root length, SL = shoot length, SV = seedling vigor index, DW = dry biomass.

**Table 2:** Phytotoxic effect of aqueous plant extracts of Fabaceae plants on germination and seedling growth of different broadleaved weed species.

Treatments	GP (%)	T_50_ (days)	GE	GI	RL (cm)	SL (cm)	SVI	DW (mg)
***T*. *portulacastrum***								
**DWTC**	73.75 a	4.00 b	35.00 a	16.02 a	2.57 a	4.05 a	488.88 a	8.25 a
***C*. *occidentalis***	57.50 b	6.16 a	12.50 b	7.91 b	0.82 c	1.91 b	155.00 b	2.45 c
***S*. *sesban***	40.00 c	4.47 ab	13.75 b	9.30 b	1.32 b	2.07 b	136.13 b	4.27 b
***M*. *alba***	31.25 d	4.21 b	16.25 b	11.32 b	0.92 c	1.57 c	87.62 c	1.55 d
**LSD**	5.66	2.01	12.2	3.46	0.22	0.24	29.91	0.81
**SE**	2.6021	0.9251	5.6366	1.5888	0.1021	0.1141	13.730	0.3718
***P*. *hysterophorus***								
**DWTC**	63.75 a	2.64	42.50 a	25.77 a	1.44 a	2.80 a	269.50 a	8.67
***C*. *occidentalis***	30.00 b	3.58	23.75 b	13.86 b	1.10 b	1.74 b	86.41 b	3.92
***S*. *sesban***	6.25 c	1.87	5.00 c	2.25 c	0.92 b	1.13 c	12.63 c	4.50
***M*. *alba***	28.75 b	3.16	8.75 c	6.52 c	1.11 b	1.36 bc	67.97 bc	6.62
**LSD**	14.38	NS	11.00	6.27	0.25	0.43	68.16	NS
**SE**	7.192	1.7475	5.0518	2.8779	0.1147	0.1985	31.283	3.19
***R*. *dentatus***								
**DWTC**	67.50 a	2.62 b	36.25 a	19.54 a	1.77 a	2.60 a	296.25 a	8.02 a
***C*. *occidentalis***	26.2 d	4.18 a	16.25 b	8.20 c	1.32 c	1.90 b	85.00 c	2.30 c
***S*. *sesban***	36.25 c	2.79 b	23.75 b	12.62 b	1.57 b	1.92 b	126.63 b	4.25 b
***M*. *alba***	55.0 b	3.83 ab	41.25 a	19.42 a	1.18 d	1.40 c	141.76 b	7.27 a
**LSD**	8.46	1.37	9.16	3.35	0.09	0.42	40.02	0.93
**SE**	3.8864	0.6302	4.2081	1.5389	0.0441	0.1945	18.372	0.4274
***M*. *indica***								
**DWTC**	62.50 a	3.00 b	13.75	11.72 a	10.31	2.54 a	356.25 a	6.67 a
***C*. *occidentalis***	10.8 c	8.25 a	7.50	3.35 c	1.97	1.31 b	77.32 c	1.32 c
***S*. *sesban***	0.00 d	NG	NG	NG	NG	NG	NG	NG
***M*. *alba***	22.50 b	5.87 a	11.25	6.35 b	3.15	1.67 b	183.55 b	2.90 b
**LSD 5%**	10.75	1.31	NS	3.00	NS	0.52	94.18	0.58

Means having similar letters do not differ significantly at 5% probability, NS = Non-significant, DWTC = Distilled water treated control, GP = germination percentage, T_50_ = time to 50% germination, GE = germination energy, GI = germination index, RL = root length, SL = shoot length, SV = seedling vigor index, DW = dry biomass.

Aqueous extracts of *C*. *occidentalis* significant delayed time to 50% germination of *T*. *portulacastrum* and *M*. *indica*. Germination energy of *T*. *portulacastrum* was significantly reduced by all plant extracts, while *M*. *indica* remained unaffected (Table 2). All plant extracts significantly reduced (15–50%) germination index of *T*. *portulacastrum* as compared to DWTC. The *S*. *sesban* and *M*. *alba* extracts caused least reduction (2.25 and 6.25) in germination index of *P*. *hysterophorus*.

The *C*. *occidentalis* and *M*. *alba* extracts resulted in the lower root length of *T*. *portulacastrum* (0.82 cm and 0.92 cm, respectively) and *M*. *indica* (1.97 and 3.15 cm, respectively). All extracts caused significant reduction in root length (1.10, 1.11 and 0.92 cm) of *P*. *hysterophorus*. As compared to DWTC, *M*. *alba* extract caused the highest reduction (61% and 40%) in shoot length of *T*. *portulacastrum* and *R*. *dentatus*, whereas *S*. *sesban* extract resulted in the lowest shoot length (1.13 cm) in *P*. *hysterophorus* (Table 2).

The least value of seedling vigor index (87.62) *T*. *portulacastrum* was recorded in response to *M*. *alba* extract, while *S*. *sesban* extract resulted in the lowest value (12.63) of seedling vigor index in *P*. *hysterophorus*. However, *C*. *occidentalis* extract resulted in the lowest seedling vigor index of *R*. *dentatus* (85.00) and *M*. *indica* (77.32). The *M*. *alba* extract resulted in the lowest dry weight (1.55 mg) of *T*. *portulacastrum*, while *C*. *occidentalis* extract resulted in the lowest dry weights (2.30 mg and 1.32 mg) of *R*. *dentatus* and *M*. *indica*, respectively.

Data relating to pot experiment is given in Tables 3 and 4. Applied extracts significantly altered the biomass and chlorophyll contents of studied weed species in pot experiment (Table 3). The lowest chlorophyll content (8.4) in *T*. *portulacastrum* with foliar application of *C*. *occidentalis* extract, whereas the contents were *P*. *hysterophorus* (21.02), *R*. *dentatus* (8.70) and *M*. *indica* (22.0) with the application of *M*. *alba* extract. Statistically similar values of chlorophyll contents in *P*. *hysterophorus* and *R*. *dentatus* were observed with the application of *S*. *sesban* and *C*. *occidentalis* extracts, respectively (Table 4).

**Table 3:** Analysis of variance (mean squares) of phytotoxic effect of aqueous plant extracts of Fabaceae plants on germination and seedling growth of different broadleaved weed species.

SOV	DF	GP	T_50_	GE	GI	RL	SL	SVI	DW
***T*. *portulacastrum***									
**Treatment**	3	1427.0***	3.62	443.7	50.15*	2.58***	4.48***	134718***	32.70***
**Error**	12	13.54	1.71	63.54	5.04	0.02	0.02	377	0.276
**Total**	15								
***P*. *hysterophorus***									
**Treatment**	3	2247.4**	2.16	1162.5***	424.3***	0.186***	2.18***	49652.2***	18.77
**Error**	12	250.5	6.10	51.04	16.56	0.026	0.078	1957.3	20.43
**Total**	15								
***R*. *dentatus***									
**Treatment**	3	1370.8***	2.36*	522.9***	122.7***	0.274***	0.970***	34149.8***	28.43***
**Error**	12	30.21	0.79	35.4	4.73	0.003	0.075	675.1	0.3654
**Total**	15								
***M*. *indica***									
**Treatment**	3	3008.3***	46.51***	143.7***	98.88***	80.82***	4.46***	97359.0***	33.35***
**Error**	12	91.67	0.723	17.70	3.80	57.72	0.115	3737.4	0.1413
**Total**	15								

SOV = source of variation

* = Significant, DF = degree of freedom, GP = germination percentage, T_50_ = time to 50% germination, GE = germination energy, GI = germination index, RL = root length, SL = shoot length, SV = seedling vigor index, DW = dry biomass.

**Table 4:** Phytotoxic effect of aqueous plant extracts of Fabaceae plants on germination and seedling growth of different broadleaved weed species.

Treatments	Chlorophyll contents (SPAD values)	Root length (cm)	Shoot length (cm)	Seedling dry weight (mg)	Seedling leaf area (cm^2^)
***T*. *portulacastrum***					
**DWTC**	19.3 a	6.90 a	6.30 a	145.0 a	283.9 a
***C*. *occidentalis***	8.4 c	3.07 c	3.05 c	49.0 d	122.6 c
***S*. *sesban***	9.8 b	4.37 b	3.68 b	113.0 b	145.6 b
***M*. *alba***	10.0 b	4.17 b	3.81 b	81.0 c	160.4 b
**LSD**	1.25	1.05	0.54	15.91	15.28
**SE**	0.5779	0.4857	0.2524	7.3030	7.0134
***P*. *hysterophorus***					
**DWTC**	30.1 a	4.96 a	3.70 a	56.5 a	751.6 a
***C*. *occidentalis***	25.4 b	3.76 b	3.21 ab	48.5 b	403.8 c
***S*. *sesban***	23.6 bc	4.10 b	2.81 b	33.2 c	627.5 b
***M*. *alba***	21.0 c	2.63 c	2.13 c	25.7 d	171.3 d
**LSD**	3.46	0.62	0.67	7.48	116.23
**SE**	1.5909	0.2862	0.3096	3.4369	53.345
***R*. *dentatus***					
**DWTC**	13.6 a	6.27 a	10.92 a	80.5 a	536.0 a
***C*. *occidentalis***	9.6 bc	3.09 c	4.87 bc	29.0 bc	276.3 c
***S*. *sesban***	10.4 b	4.09 b	5.70 b	33.2 b	360.0 b
***M*. *alba***	8.7 c	2.64 c	3.62 c	25.0 c	187.3 d
**LSD**	1.43	0.49	1.94	7.35	68.85
**SE**	0.6569	0.2263	6.8597	3.3773	31.600
***M*. *indica***					
**DWTC**	37.4 a	9.67 a	9.57 a	53.7 a	611.0 a
***C*. *occidentalis***	28.3 b	6.40 c	7.22 b	33.5 b	204.4 b
***S*. *sesban***	33.2 a	7.88 b	6.68 b	31.7 b	152.5 c
***M*. *alba***	22.0 c	4.77 d	5.0 c	10.2 c	61.3 d
**LSD 5%**	4.43	1.27	0.70	13.09	46.87

Means having similar letters do not differ significantly at 5% probability, DWTC = Distilled water treated control.

The lowest root lengths were recorded for *T*. *portulacastrum* (3.07 cm) with *C*. *occidentalis* extract. The lowest root length of *R*. *dentatus* (2.64 cm and 3.09 cm) was recorded in response to *M*. *alba* and *C*. *occidentalis* extracts, respectively. The *C*. *occidentalis* extract caused the highest reduction (50%) in shoot length of *T*. *portulacastrum*, while *M*. *alba* in shoot lengths of *P*. *hysterophorus* (42%) and *M*. *indica* (47%) as compared to DWTC. However, both *C*. *occidentalis* and *M*. *alba* extracts produced lower values of shoot lengths (3.62 and 4.87 cm) in *M*. *indica* seedlings. Foliar application of *C*. *occidentalis* extract resulted in the lowest dry weight (49 mg) of *T*. *portulacastrum* seedlings. Data indicated that *C*. *occidentalis* extract resulted in the lowest leaf area (122.6 cm^2^) of *T*. *portulacastrum*, while *S*. *sesban* extract in the lowest leaf areas of *P*. *hysterophorus* (171.3 cm^2^), *R*. *dentatus* (187.3 cm^2^) and *M*. *indica* (61.3 cm^2^) (Table 4).

## Discussion

Soon valley is known as central salt range, located in the north-west side of the district Khushab, and has rich floristic diversity. The plants naturally found here have significant medicinal value [51,52]. Abbas et al. [53] revealed that plants of this valley are the richest source of biologically active components such as steroids, phytolipids, alkaloids, phenolics and antimicrobial agents. There are some Fabaceae plants which are abundantly distributed here. These include *Cassia occidentalis* (coffee senna), *Sesbania sesban* (Egyptian river hemp) and *Melilotus alba* (Yellow sweet clover). Fabaceae synthesize greater diversity of secondary metabolites compared to other plant families [54]. These include alkaloids and amines, non-protein amino acids, cyanogenic glucosides, and peptides [54].

The *C*. *occidentalis* is a well-known medicinal plant, rich in fedegoso that contains minute amount of anthraquinones that gives it substantial purgative and laxative properties [55]. In addition, fedegoso contains other secondary metabolites such as achrosine, aloe-emodin, anthrones, apigenin, aurantiobtusin, campesterol, cassiollin, chryso-obtusin, chrysophanic acid, chrysarobin, chrysophanol, chrysoeriol, emodin, essential oils, funiculosin, galactopyranosyl, helminthosporin, islandicin, kaempferol, lignoceric acid, linoleic acid, linolenic acid, mannitol, mannopyranosyl, matteucinol, obtusifolin, obtusin, oleic acid, physcion, quercetin, rhamnosides, rhein, rubrofusarin, sitosterols, tannins, and xanthorin. The *S*. *sesban* is a commonly used leguminous fodder as well as valuable green manure crop. It contains one of the toxic non-protein amino acids that is called canavanine [56]. The *M*. *alba* is considered highly allelopathic. Various allelochemicals, including the highest quantity of coumarin content followed by coumarin, flavonoids, phenolic acids, triterpenes and saponins are found in *M*. *alba* [57–59].

Initial screening indicated that aqueous extracts of all plants were more phytotoxic against lettuce. The possible reasoning of higher allelopathic activity of aqueous extracts in comparison to their N-hexane fractions seems to be the higher concentrations of water soluble phenolics that caused more inhibitory effect [60–62]. Tanveer et al. [42] and Safdar et al. [43] revealed that aqueous extracts of *Euphorbia dracunculoides*, *Dicliptera bupleuroides* and *Justicia adhatoda* exhibited greater allelopathic activity than their organic solvents (n-hexane, chloroform, ethylacetate, 1-butanol) against germination and seedling growth of chickpea, wheat and broadleaved weeds, respectively. Our observations are supported by Oudhia & Tripathi [63] and Sahid & Sugau [64] who reported significant inhibitory effect of *Lantana camara* aqueous extracts on germination and seedling growth of *T*. *aestivum* and many vegetable species. Oyun et al. [65] demonstrated that aqueous extracts derived from leaves of *Gliricidia sepium* and *Acacia auriculiformis* had pronounced phyto-inhibitory effect on germination and seedling vigor of maize. Wakjira et al. [66] stated that aqueous extract of *P*. *hysterophorus* significantly inhibited germination index of lettuce. Tanveer et al. [67] also reported that aqueous extract of *Achyranthes aspera* significantly inhibited germination index of *Sorghum bicolor*.

In Petri dish germination bioassay, differential phyto-inhibitory effect on germination and seedling growth of different weed species were observed in response to aqueous extracts of different plants. The highest reduction in germination percentage of *T*. *portulacastrum* and *R*. *dentatus* was noted with *M*. *alba* and *C*. *occidentalis* extracts. Similarly, *S*. *seban* extract reduced the germination percentage of *P*. *hysterophorus* and *M*. *indica* by 90% and 100%, respectively. The reduction in germination percentage of weeds might be the result of presence of phytotoxic compounds that limited the underlying germination processes. Our results are supported by Randhawa et al. [68] who reported reduced germination percentage of *T*. *portulacastrum* in response to sorghum water-soluble extract. Delayed germination of weeds by application of plant extracts was attributed to their phyto-inhibitory effect that hindered germination process. Our results are supported by Mubeen et al. [69] who observed that aqueous extracts of different weeds showed significant reduction in time to 50% germination of *Oryza sativa*.

The decrease in shoot lengths of weeds seems to be the phyto-inhibitory effect of allelochemicals in these extracts. Our results are supported by Safdar et al. [70] who observed significant reduction in maize shoot length in response to aqueous extracts of *A*. *aspera* and *P*. *hysterophorus*. The decreased seedling vigor index is the result of reduced germination percentages and seedling lengths. The reduction in dry weight might be attributed to reduced root and shoot growth due to the presence of toxic compounds in studied extracts. These results are supported by Komal [71] who observed significant allelopathic effect of foliar extracts of C. *occidentalis* on dry weight of maize. The reduction in leaf area of weeds in response to foliar application of plant extracts seems to be the consequence of lower shoot growth and chlorophyll content. These results are supported by Musyimi et al. [72] who reported that application of *Sesbania sesban* (L.) Merrill extract significantly influenced the leaf area of *Solanum nigrum* L.

## Conclusions

The *M*. *alba*, *S*. *sesban* and *C*. *occidentalis* extracts showed higher phytotoxicity against seed germination of *T*. *portulacastrum*, *P*. *hysterophorus*, *M*. *indica* and *R*. *dentatus*. Similarly, application of *C*. *occidentalis* on the seedlings had the highest inhibitory effect on *T*. *portulacastrum*, and *M*. *alba* against *P*. *hysterophorus*. Hence, these extracts cab ne recommend for the management of these weed species. However, their thorough understanding under field conditions is necessary before making a general recommendation.

## Supporting information

S1 Dataset (XLSX)
